# Ubenimex Combined with Pemetrexed Upregulates SOCS1 to Inhibit Lung Adenocarcinoma Progression via the JAK2-STAT3 Signaling Pathway

**DOI:** 10.1155/2022/5614939

**Published:** 2022-06-25

**Authors:** Quan Chen, Bingbing Wu, Pengfei Ge, Peng Zhang, Xia Chen

**Affiliations:** Department of Thoracic Surgery, Hospital Affiliated 5 to Nantong University (Taizhou People's Hospital), Taizhou 225300, China

## Abstract

To study the effects of ubenimex (UBE) combined with pemetrexed (PEM) on lung adenocarcinoma cell behavior and its molecular mechanism, the tissue samples from lung adenocarcinoma patients who received PEM chemotherapy, those with PEM combined with UBE chemotherapy, and healthy volunteers were retrieved and analyzed. The expression levels of the suppressor of cytokine signaling 1 (SOCS1) in the human lung adenocarcinoma cancer cell lines A549 and PC-9 and tissues were detected by qRT-PCR. MTT assay was performed for cell proliferation. Cell apoptosis was detected by flow cytometry. Cell invasion ability was assessed using the Transwell assay. The expression levels of the JAK2/STAT3 signaling pathway proteins and apoptosis-related proteins were detected by Western blot. The antitumor effect of PEM combined with UBE was tested in nude mice using the tumor formation assay. Our results showed that UBE treatment, alone or combined with PEM, inhibited lung adenocarcinoma cell migration, invasion, and proliferation; promoted apoptosis; significantly increased the G0/G1-phase cell ratio; reduced the S-phase cell ratio; and inhibited the *in vivo* growth of tumor cells. UBE alone or in combination with PEM also inhibited the JAK2/STAT3 signaling pathway in lung adenocarcinoma cells. In addition, UBE combined with PEM therapy was associated with increased SOCS1 expression in patients' serum and knocking down SOCS1 reversed the antitumor effects of UBE and PEM. Overall, combination therapy with UBE and PEM could inhibit the JAK2-STAT3 signaling pathway by upregulating SOCS1 expression to hinder the progression of lung adenocarcinoma cells.

## 1. Introduction

Lung cancer has one of the highest mortality rates and extremely poor prognoses among all malignant tumors. It is associated with the death of nearly 1.5 million people annually [1–3]. About 85% of patients with advanced lung cancer are not eligible for curative surgery because, by the time of clinical diagnosis, most lung cancer has already reached an advanced stage, which is one of the main factors for the high mortality rate of lung cancer. Based on its histological characteristics, lung cancer can be divided into 2 subtypes: non-small cell lung cancer (NSCLC) and small cell lung cancer (SCLC). SCLC consists of ~15% of all lung cancer cases and accounts for ~85% of all NSCLC [4]. Further, NSCLC can be divided into 3 primary histological subtypes: large cell carcinoma, lung squamous cell carcinoma (LUSC), and lung adenocarcinoma (LUAD). Despite the significant progress made in the treatment of NSCLC, its recurrence rate is still very high [5, 6]. Therefore, to improve the outcomes of NSCLC treatment, the urgent need to formulate new therapeutic drugs to improve patients' survival rates has become a current research hotspot.

At present, the most commonly used clinical treatment plan is systemic chemotherapy based on platinum compounds combined with adjuvant drug therapy after chemotherapy to enhance therapeutic effects [7]. A significant number of studies have shown that platinum-based drugs combined with pemetrexed (PEM) were well bore in NSCLC patients and extended their overall survival and are now recommended as first-line treatment in lung adenocarcinoma [8, 9]. However, in other studies, platinum substances were found to have negative effects such as nephrotoxicity, sepsis, and neurotoxicity with serious drug resistance [10].

Ubenimex (UBE), also known as bestatin, has the chemical name of N-[(2S,3R)-3-amino-2-hydroxy-4-phenylbutyryl]-L leucine and was marketed in Japan in 1987 as an aminopeptidase N (APN) inhibitor [11]. It was shown to improve immunocompetent cell functions and had antitumor effects and has often been used as an auxiliary drug for anticancer treatments in gastric cancer, bladder cancer, and ovarian cancer [12]. It has now been demonstrated that UBE inhibits hepatocellular carcinoma tumor growth *in vivo* in synergy with PEM and enhances its drug sensitivity [13]. However, there are no reports on the treatment effects of UBE combined with PEM on lung adenocarcinoma nor its mechanism of action. This study is aimed at examining the impacts of UBE on the invasion, apoptosis, proliferation, migration, and cell cycle of lung adenocarcinoma cells and investigating its possible underlying mechanism.

## 2. Materials and Methods

### 2.1. Specimens

The sera of lung adenocarcinoma patients (*n* = 40) (before treatment and 1 week after chemotherapy) who underwent PEM (500 mg/m^2^ at 3-week intervals) chemotherapy (PEM group, *n* = 20) and combined treatment with PEM and UBE (PEM + UBE group; UBE 30 mg per day) were collected. Diagnoses were based on pathological evidence.

The serum of healthy volunteers (*n* = 20) undergoing physical examination at the hospital during the same period was also collected and used as the control group (HC group). All participants provided written consent for the anonymous use of their data for research purposes, and the study was approved by the Ethics Committee of the Hospital Affiliated 5 to Nantong University (Taizhou People's Hospital, Taizhou, China).

### 2.2. Cell Culture and Treatment

Human lung adenocarcinoma cancer cell lines PC-9 and A549 were acquired from the Shanghai Institute of Cell Research, China. All cells were cultured in a high-sugar DMEM culture medium with 10% fetal bovine serum (FBS) (Invitrogen, USA) and 1% penicillin-streptomycin. They were kept in an incubator at 37°C with 5% CO_2_ and a humidity of 95%.

Cells in the logarithmic growth phase were collected, diluted to 2 × 10^6^ cells/ml, and seeded in a 6-well plate. Intervention and transfection were performed when the cells were cultured to a confluence of 80% to 90%. The cells were divided into the following groups based on the treatment provided: sham group, 0.1 mg/ml UBE group, 0.5 mg/ml UBE group, 1 mg/ml UBE group, and 1 mg/ml UBE + 100 nM PEM group. The cell transfection groups were as follows: the shNC group, UBE (1 mg/ml) + PEM (100 nM) + shNC group, and UBE + PEM + sh-SOCS1 group. Transfection was performed using the corresponding transfection kit instructions, and the cells were collected 48 hours after transfection.

### 2.3. Establishment of the Tumor Xenograft Model

Fifteen adult BALB/c female nude mice (age, 4 weeks) were subcutaneously injected with 3 × 10^6^ A549 cells in 150 *μ*l PBS at their right axilla. When the tumor volume had reached a median size about 100 mm^3^ [14], the mice were randomly divided into 5 groups: (1) sham group: intraperitoneal injection with physiological saline; (2) 5 mg/ml UBE group: intraperitoneal injection with 5 mg/ml ubenimex; (3) 10 mg/ml UBE group: intraperitoneal injection with 10 mg/ml ubenimex; (4) 15 mg/ml UBE group: intraperitoneal injection with 15 mg/ml ubenimex; and (5) UBE + PEM group: intraperitoneal injection with 15 mg/ml ubenimex and 150 mg/ml pemetrexed. After 21 days of continuous treatment, the tumor tissues were removed and weighed and their length and width were measured to determine the tumor volume.

### 2.4. Real-Time Quantitative Polymerase Chain Reaction (qRT-PCR)

Serum and cells were collected, and the total RNA extraction kit was used to extract total cellular RNA before storage at −80°C. Then, reverse synthesizes of cDNA were performed following a reverse transcription PCR kit protocol. The concentration and purity of the resulting cDNA were then tested. The cDNA was taken and synthesized SOCS1 mRNA following real-time PCR instructions, using the following reaction procedures: 95°C for 1 min; 95°C for 40 s, 58°C for 40 s, and 72°C for 45 s for 35 cycles, and 72°C for 10 min. Data analysis was performed with the 2^−ΔΔ*Ct*^ method [13]. The primer sequences used are shown in Table 1.

### 2.5. MTT (3-[4,5-Dimethylthiazol-2-yl]-2,5 Diphenyl Tetrazolium Bromide) Assay to Determine the Cell Proliferation Rate

The transfected PC-9 or A549 cells were collected. The digestion of cells was performed using trypsin, and the concentration of the cells was altered to 1 × 10^4^ cells/ml and inoculated into 96-well plates, and MTT assays were conducted after 24, 48, and 72 h of culture. 20 *μ*l of MTT solution (5 mg/ml) was added to the wells for a 4-hour incubation. Discard the supernatant and replenish 150 *μ*l DMSO, mixed at room temperature (RT) for 5 minutes, and then the absorbance was evaluated with a microplate reader at 490 nm.

### 2.6. Detection of Apoptosis by Flow Cytometry

An apoptosis detection kit was used to detect cell apoptosis. The Falcon test tube was taken, and the negative control tube and the sample tube number were programmed according to the order of the specimen. PBS was used to wash the cells to make a suspension of 1 × 10^6^ cells/ml with a buffer. 100 *μ*l of the cell suspension was supplemented to the Falcon test tube, followed by nucleic acid dye and annexin V, which were then placed in a dark place at room temperature for 15 minutes. The annexin V-biotin reagent was then used for detection, to which PI was added and placed in a dark place for 15 minutes at RT. 400 *μ*l of 1x binding buffer was included in each test tube, and within 1 hour, the FACScanflow Cell flow cytometry system (Becton Dickinson, San Diego, CA, USA) was used to measure the results.

### 2.7. Cell Migration and Invasion Ability Detected by Transwell Assay

#### 2.7.1. Invasion Assay

Matrigel was removed from −20°C and placed at 4°C overnight to become liquid. Matrigel was diluted with a serum-free medium at 4°C at a ratio of 1 : 6. 100 *μ*l which was put into the upper Transwell chamber and placed at 37°C for 3–5 hours to turn into a solid state. The following steps were the same as those in the migration assay. 100 *μ*l of cells was placed into the upper chamber, and 500 *μ*l of 10% FBS medium was placed in the lower layer. The cells were cultured for 24 hours, fixed, stained, and counted.

#### 2.7.2. Migration Assay

The transfected cells were cultured to the logarithmic growth phase, the cells were collected, serum-free DMEM medium containing 10 g/L BSA was added, and the cell concentration was diluted to 2 × 10^5^ cells/ml after 12 hours of starvation culture. 500 *μ*l of 10% FBS medium was supplemented as migration chemokines to the lower culture well of Transwell. 100 *μ*l of diluted cells was placed into the upper chamber of Transwell and incubated in a 37°C with 5% CO_2_ for 24 h. Nonmigrated cells and Matrigel in the upper chamber were cleaned off using a cotton swab, and the cells were fixed with ice formaldehyde and observed by crystal violet staining.

### 2.8. Western Blot

RIPA lysate was applied to lyse the cells of each group for 20 min, and the cells were disrupted by ice bath ultrasonication. The proteins were then collected, and their concentration was detected. SDS-PAGE was performed, transported to PVDF membrane, and blocked at RT for 1 h. Primary antibodies, GAPDH, cyclinb1, Bax, p-JAK2, SOCS1, JAK2, STAT3, p-STAT3, and Bcl-2 were added and incubated overnight at 4°C. The membrane was rinsed twice, added with the diluted enzyme-labeled secondary antibody, and incubated at RT for 1 h. Protein levels were analyzed using GAPDH as an internal reference.

### 2.9. Immunohistochemistry Experiment

The mice tumor tissues were excised on day 21 of treatments. They were fixed with formaldehyde and embedded in paraffin. They were baked at 60°C for 20 minutes and placed in xylene solution, which was changed and soaked for 15 minutes each. Ethanol was then used to dehydrate according to laddered concentrations. The slides were washed, and 3% H_2_O_2_ was added to each slice and placed at RT to soak for 25 min. Citric acid buffer was added and cooked in a microwave oven for 3 minutes, and the antigen retrieval solution was dropped on, placed at RT for 10 minutes, and cleaned with PBS. Normal goat serum blocking solution was added for 30 min at RT. Then, diluted primary antibodies were added and incubated at 4°C overnight. The tissues were washed 3 times in PBS before goat anti-rabbit IgG secondary antibody was added and incubated for 30 min. SABC was added and kept in a 37°C incubator for 30 min. The chromogenic reagent was added for color development, stained in hematoxylin after washing, and dehydrated accordingly to laddered ethanol concentrations. They were then immersed in transparent xylene and sealed with neutral resin, and an upright microscope was used to assess the slides.

### 2.10. Statistical Analysis

The experimental data were analyzed using the SPSS 21.0 software. The *t*-test was used between the two groups, and the single-factor analysis of variance was applied for multiple group comparison. Mean ± standard error (SED) was employed for result expression, and *P* < 0.05 was regarded as statistically significant.

## 3. Results

### 3.1. UBE Combined with PEM Treatment Promotes the Expression of SOCS1 in Patients' Serum

Before chemotherapy, the expression levels of SOCS1 in the patients' serum of the two treatment groups were drastically reduced compared with the HC group (*P* < 0.05) and no considerable difference was observed between the PEM and UBE + PEM group (*P* > 0.05) (Figure 1). After chemotherapy, although the expression levels of SOCS1 in the serum of patients from the UBE + PEM groups were significantly higher than before chemotherapy (*P* < 0.05) (Figure 1), they were still lower than those of the HC group. In addition, we also observed that the expression level of SOCS1 in the UBE + PEM group was significantly higher than that in the PEM group (*P* < 0.05).

### 3.2. UBE Treatment Alone or Combined with PEM Inhibits the Migration, Invasion, and Proliferation of Lung Adenocarcinoma Cells

Compared with the sham group, the proliferation rate, migration ability, and invasion ability of PC-9 and A549 cells in the three UBE treatment groups and UBE + PEM group were substantially reduced (*P* < 0.05), in a concentration-dependent manner (Figures 2(a)–2(c)). Also, compared with those of the 1 mg/ml UBE group, the cell migration ability, invasion ability, and proliferation rate of the UBE + PEM group were significantly lower (*P* < 0.05).

### 3.3. Effects of UBE Treatment Alone or Combined with PEM on Apoptosis and Cell Cycle of Lung Adenocarcinoma Cells

Here, we observed that the apoptotic rates of cells in the two UBE treatment groups (UBE, 0.5 and 1 mg/ml) and the UBE + PEM group were considerably enhanced compared with those in the sham group (*P* < 0.05) (Figures 3(a) and 3(b)). The G0/G1-phase cell ratio was amplified, while that of the S-phase cell proportion was reduced. Western blot analysis showed that cyclinb1 and Bcl-2 expression levels in the cells were drastically lessened, while those of Bax were significantly enhanced (*P* < 0.05) and were concentration dependent, compared with those of the sham group (Figure 3(c)).

In regard to the different types of UBBE treatment, compared with that of the 1 mg/ml UBE group, the cell apoptosis rate of the UBE + PEM group was significantly amplified (*P* < 0.05), its G0/G1-phase cell proportion was considerably enhanced, and its S-phase cell proportion was significantly lowered (Figures 3(a) and 3(b)). Further, the expression levels of cyclinb1 and Bcl-2 were significantly lowered, and those of Bax were significantly increased in the UBE + PEM group compared with the 1 mg/ml UBE group (Figure 3(c)).

### 3.4. Treatment with UBE Alone or in Combination with PEM Can Inhibit the JAK2/STAT3 Signaling Pathway of Lung Adenocarcinoma Cells

Mechanistically, Western blot experiments showed that compared with those of the sham group, the expression levels of SOCS1 in the cells of the two UBE treatment groups (0.5 and 1 mg/ml UBE) and UBE + PEM group were significantly increased (*P* < 0.05), while the expression levels of p-JAK2 and p-STAT3 expression and the ratio of p-JAK2/JAK2, p-STAT3/STAT3 were significantly decreased (*P* < 0.05). STAT3 and JAK2 expression levels were not significantly different between the treatment and no treatment groups (*P* > 0.05).

Further, we also observed that, compared with those of the 1 mg/ml UBE group, the SOCS1 expression levels in cells of the UBE + PEM group were significantly increased (*P* < 0.05), while the expression levels of p-JAK2 and p-STAT3 expression and the ratio of p-JAK2/JAK2, p-STAT3/STAT3 were significantly decreased (*P* < 0.05). No difference in STAT3 and JAK2 expression levels between the treatment groups was observed (*P* > 0.05) (Figures 4(a)–4(d)).

### 3.5. Knockdown of SOCS1 Reversed the Antitumor Effects of UBE and PEM

First, we assessed the levels of SOCS1 using treatments and no treatment in the lung cancer cells. qRT-PCR analysis showed that the SOCS1 expression level in the cells of the 2 UBE treatment groups and UBE + PEM group was significantly enhanced and was concentration dependent compared with that of the sham group (*P* < 0.05) (Figure 5(a)). Also, compared with the 1 mg/ml UBE group, the SOCS1 expression levels in the UBE + PEM group were markedly higher (*P* < 0.05), while a significant difference was seen between the sham group and the 0.1 mg/ml UBE group (*P* > 0.05) (Figure 5(a)).

Next, we knocked down SOCS1 in the cancer cell lines. The results demonstrated that compared with the shNC nontreatment group, the cell proliferation, invasion, and migration ability of the UBE + PEM + shNC group were significantly reduced (Figures 5(b)–5(d)), their apoptosis rate and G0/G1-phase cell ratio were significantly increased (Figures 5(e) and 5(f)), and their S-phase cell ratio was reduced (*P* < 0.05). Further, compared with the UBE + PEM + shNC group (expression of SOCS1 was not knocked down), the cell proliferation, invasion, and migration ability of the UBE + PEM + sh-SOCS1 group were significantly increased (Figures 5(b)–5(d)), their apoptotic rate and G0/G1-phase cell ratio were significantly reduced (Figures 5(e) and 5(f)), and their S-phase cell ratio was increased.

Mechanistically, compared with the shNC nontreatment group, in the UBE + PEM + shNC group, the expression levels of Bcl-2 and Cyclinb1 in cells were significantly reduced (*P* < 0.05), Bax and SOCS1 expression levels were significantly increased (*P* < 0.05), and p-JAK2/JAK2 and p-STAT3/STAT3 ratios were significantly decreased. In addition, compared with the UBE + PEM + shNC group, in the UBE + PEM + sh-SOCS1 group, the expression levels of Bcl-2, cyclinb1, and the ratio of p-JAK2/JAK2, p-STAT3/STAT3 in cells were significantly increased (*P* < 0.05), while Bax and SOCS1 expression levels were significantly decreased (*P* < 0.05) (Figures 5(g) and 5(h)).

### 3.6. Ubenimex Combined with Pemetrexed Treatment Inhibits Tumor Growth *In Vivo*

Here, we investigated the effects of UBE and PME in nude mice. The results showed that compared with the sham group, the SOCS1 expression levels in mice tumor tissues of the three UBE treatment groups and the UBE + PEM group were significantly increased (*P* < 0.05) and were concentration dependent (Figure 6(a)). Further, compared with the 15 mg/ml UBE group, the SOCS1 expression level in the UBE + PEM group was significantly enhanced (*P* < 0.05). The results of tumor formation experiments in nude mice showed that the combined treatment of UBE and PEM was associated with a significant reduction in tumor volume and weight and demonstrated better antitumor effects than UBE treatment alone (*P* < 0.05) (Figure 6(b)–6(d)). Additionally, when compared with those of the sham group, the expression levels of Ki67 in the tumor tissues of the 3 UBE treatment groups and UBE + PEM group were significantly decreased (*P* < 0.05) and the expression levels of Ki67 in tumor tissues of the UBE + PEM group were considerably lower than those of the 15 mg/ml UBE group (*P* < 0.05) (Figure 6(e)).

## 4. Discussion

Although there are multiple treatments recommended for NSCLC, chemotherapy remains the main treatment modality [15]. With respect to chemotherapy, pemetrexed is considered the preferred drug for advanced NSCLC, both as neoadjuvant and adjuvant therapy due to its favorable therapeutic benefit [16, 17], even in patients with brain metastases [18]. Ubenimex is an APN inhibitor that can inhibit APN expression in human ovarian cancer cells. APN has a critical role in controlling the differentiation and growth of cancer cells [19]. Inhibiting the expression or activity of APN has been attributed to a reduction in the migration, invasion, and proliferation of many types of cells [20], such as human clear cell ovarian carcinoma cells [21], human malignant melanoma cells, and human skin cancer cells [22]. Given that UBE enhances the tumor suppressive effect of PEM [13], in this study, we investigated the combined effect of these two drugs on lung adenocarcinoma. This study found that ubenimex alone or combined with PEM inhibited the migration, invasion, and proliferation of lung adenocarcinoma cells and the inhibitory effect gradually increased with an increase in drug concentration.

The growth of tumors depends on the apoptosis and proliferation of tumor cells, and by inducing cell cycle arrest and promoting cell apoptosis, these effects can be achieved [23]. Ubenimex was shown to stimulate G2/M cell cycle arrest in glioma cells [24]. Cycle-related proteins are key in regulating the cell cycle processes. CyclinB1 is a key G2/M-phase cycle checkpoint protein participating in the transformation of G2/M-phase cells, promoting cells to enter the M phase and ensuring normal mitosis progress. When cyclinB1 protein expression is reduced, the tumor cells can be seized in the G2/M phase to inhibit cell proliferation [25]. This study found that treatment with ubenimex alone or in combination with pemetrexed led to a significant increase in G0/G1-phase lung adenocarcinoma cells, a noteworthy decline in S-phase cells, and a considerable decline in cyclinB1 protein expression levels, which in turn could inhibit cell proliferation.

In addition, flow cytometry analysis showed that the treatment of ubenimex combined with pemetrexed was associated with an increase in the early apoptosis rate of lung adenocarcinoma cells and induced cell apoptosis. Apoptosis is an active cell death process, and it is also an important control mechanism that determines whether to kill cells with genetic changes that are not repaired. The entire process involves the expression of a series of related genes, including the Bcl-2 gene family, which is currently recognized as a gene closely related to apoptosis. Research has demonstrated that Bax and Bcl-2 are characteristic antiapoptotic and proapoptotic proteins of the Bcl-2 family [26]. In this study, we observed that ubenimex combined with pemetrexed treatment lowered proapoptotic proteins Bcl-2 and cyclinb1 expression levels in cells and significantly increased Bax expression levels that inhibited apoptosis. In addition, tumor formation experiments in nude mice showed that ubenimex alone or combined with pemetrexed was associated with tumor growth inhibition in *in vivo* settings. Therefore, these findings suggest that ubenimex could induce cycle arrest in lung adenocarcinoma cells, increase cell apoptosis, inhibit cell proliferation, and inhibit tumor growth by downregulating Bcl-2 and cyclinb1 and upregulating Bax to cause cell apoptosis. Also, these could be synergized with combined treatment with pemetrexed.

The Janus kinase 2/signal transducer and activator of transcription 3 (JAK2/STAT3) signal pathway is the general pathway of many cytokine signal transductions, which is broadly engaged in cell inflammation, apoptosis differentiation, and proliferation [27]. JAKs are the upstream kinases of the STATS signal transduction pathway. When activated, they induce the phosphorylation of monomeric STAT molecules in the cytoplasm to form STAT dimers and transfer them to the nucleus to adjust gene expression. The JAK/STAT signaling pathway is critical in maintaining body stability [28]. Research has demonstrated that abnormal JAK2/STAT3 signaling pathway activation occurs in lung cancer and other tumor tissues and tumor cells and it is engaged in the occurrence, metastasis, development, and invasion of tumors [29].

The SOCS family is a recently discovered class of negative regulators that can feedback and block the signal transduction process of cytokines. It can be rapidly transduced and induced by a variety of cytokines, thus constituting a negative feedback regulation of the JAK/STAT pathway which can effectively prevent the body from producing an excessive immune response and effectively prevent the progression of the disease and damage to the tissue to a certain extent [30]. The SOCS1 gene encodes a protein member of STAT inhibitors. SOCS family members are cytokine-induced negative regulators of cytokine signaling. It was originally discovered as a negative regulator of the activator of transcription STAT signaling pathway and JAK/signal transducer, and the negative regulatory effect of SOS1 on the JAK2/STAT3 signaling pathway has been confirmed [31–33]. This study showed that treatment with ubenimex alone or combined with pemetrexed could considerably increase the expression level of SOCS1 in patients' serum, lung adenocarcinoma cells, and mouse tumor tissues and inhibit the JAK2/STAT3 signaling pathway. In addition, we also found that knocking down SOCS1 could reverse the antitumor effects of UBE and PEM and trigger the JAK2/STAT3 signaling pathway. These suggest that ubenimex combined with pemetrexed in lung adenocarcinoma treatment could be therefore achieved by upregulating SOCS1 expression and then inhibiting the JAK2-STAT3 signaling pathway, further confirming the negative regulatory effect of SOS1 on the JAK2/STAT3 signaling pathway.

Despite the important findings observed in this study, there were some limitations worth mentioning. First, the clinical effectivity of ubenimex alone and in combination with pemetrexed should be further assessed in clinical trials using randomized and prospective settings. Second, in future studies, the overexpression of SOCS1 in these cells and the prognostic significance of SOCS1 in lung cancer patients should also be assessed.

## 5. Conclusion

Our findings suggest that ubenimex alone or in combination with pemetrexed could inhibit the occurrence and development of malignant biological behavior of lung adenocarcinoma cells by upregulating SOCS1 expression and then inhibiting the JAK2-STAT3 signaling pathway. These suggest ubenimex as a promising treatment for lung adenocarcinoma and SOCS1 as a new molecular target for diagnosing and treating lung adenocarcinoma.

## Figures and Tables

**Figure 1:** Comparison of SOCS1 levels in the patients' serum of each group before and after chemotherapy by qRT-PCR. ^∗^*P* < 0.05 for comparisons between the treatment groups and the HC group; ^#^*P* < 0.05 for comparison between the PEM group and the UBE + PEM group.

**Figure 2:** Effects of different types of treatments versus no treatment on the proliferation, migration, and invasion of PC-9 and A549 cells. (a) Proliferation of the cells at indicated time points under different treatments of UBE, UBE combined with PEM, and no treatment via MTT. (b) Invasion and (c) migration of the cells after 24 hours under different treatments of UBE, UBE combined with PEM, and no treatment. ^∗^*P* < 0.05 for comparison between the treatment groups and the sham group; ^#^*P* < 0.05 for comparison between the 1 mg/ml UBE group and the UBE + PEM group.

**Figure 3:** Effects of different types of treatments and no treatment on the cell cycle, apoptosis, and expression of corresponding proteins in PC-9 and A549 cells. (a) Cell cycle changes detected with flow cytometry. (b) Flow cytometry showing the apoptosis and corresponding analysis via bar charts showing the apoptosis rates in the cells. (c) Corresponding protein expression levels under different treatments and no treatments via Western blot. ^∗^*P* < 0.05 for comparison between the treatment groups and the sham group; ^#^*P* < 0.05 for comparison between the 1 mg/ml UBE group and the UBE + PEM group.

**Figure 4:** Pathway analysis based on different types of treatments and no treatment using A549 (a, b) and PC-9 (c, d) cells. (a, c) Represent the results on the Western blots, while (b, d) illustrate the relative protein expressions via histogram. ^∗^*P* < 0.05 for comparison between the treatment groups and the sham group; ^#^*P* < 0.05 for comparison between the 1 mg/ml UBE group and the UBE + PEM group.

**Figure 5:** Antitumor effects of UBE + PEM combined treatment versus no treatment in lung cancer cells with and without SOCS1 knockdown. (a) qRT-PCR detected SOCS1 expression levels in cells with and without treatments. (b) MTT detecting cell proliferation. (c) Invasion and (d) migration of the PC-9 and A549 cells without treatment (shNC), with UBE + PEM combined treatment but no SOCS1 knockdown (UBE + PEM + shNC) and with UBE + PEM combined treatment and SOCS1 knockdown (UBE + PEM + shSOCS1). (e) Flow cytometry showing the apoptosis of the shNC cells, UBE + PEM + shNC cells, and UBE + PEM + shSOCS1 cells. (f) Flow cytometry showing cell cycle changes. (g, h) Pathway analysis via Western blot of corresponding protein expression and their histogram representation of the shNC cells, UBE + PEM + shNC cells, and UBE + PEM + shSOCS1 cells. ^∗^*P* < 0.05 for comparison between the treatment groups and the sham group; ^#^*P* < 0.05 for comparison between the 1 mg/ml UBE group and the UBE + PEM group.

**Figure 6:** *In vivo* model of ubenimex combined with pemetrexed. (a) qRT-PCR detection of the SOCS1 expression levels in the tumor tissues of mice under different types of treatments. (b) Comparison of tumor volume in each group after tumor xenotransplantation in nude mice. (c) The final weight of the tumor in each group. (d) The tumor volume of each treatment group compared with no treatment. (e) Immunohistochemistry showing Ki67 expression levels in each group of mouse tumors. ^∗^*P* < 0.05 for comparison between the treatment groups and the sham group; ^#^*P* < 0.05 for comparison between the 1 mg/ml UBE group and the UBE + PEM group.

**Table 1:** qRT-PCR primer sequence.

Gene name	Primer sequence (5′-3′)
SOCS1	F-AGGCCATCTTCACGCTAAGG
	R-CCAGCTCACCTCTTTGTCTCT
GAPDH	F-TGTGTCCGTCGTGGATCTGA
	R-TTGCTGTTGAAGTCGCAGGAG

## Data Availability

The data used to support the findings of this study are included within the article. Further inquiries can be directed to the corresponding author.
